The article "Differentially Expressed Genes in Nasopharyngeal Carcinoma Tissues and Their Correlation with Recurrence and Metastasis of Nasopharyngeal Carcinoma" was retracted in 2023. Reasons: unreliable results or conclusions; concerns about the data; concerns about the peer review; concerns about the citations.

# Differentially Expressed Genes in Nasopharyngeal Carcinoma Tissues and Their Correlation with Recurrence and Metastasis of Nasopharyngeal Carcinoma

**DOI:** 10.1155/2022/1941412

**Published:** 2022-04-25

**Authors:** Haiying Yue, Huijun Zhu, Danjing Luo, Qinghua Du, Yiting Xie, Sijie Huang, Wenqi Liu

**Affiliations:** Department of Radiotherapy, The Second Affiliated Hospital of Guangxi Medical University, Nanning 530007, China

## Abstract

In this study, bioinformatics tools were used to identify key genes to study the molecular mechanism of nasopharyngeal carcinoma (NPC) development and to explore the correlation of these key genes with the recurrence and metastasis of NPC. The GSE61218 microarray dataset obtained from the Gene Expression Omnibus Database (GEO) was used. The limma R package was used to screen differentially expressed genes (DEGs) between NPC and normal nasopharyngeal (NP) tissues. KEGG functional enrichment was performed on these selected DEGs. Protein-protein interaction (PPI) networks were constructed using Cytoscape software to identify key node proteins. The NPC-metastasis microarray dataset GSE103611 was obtained from GEO to analyze the expression of DEGs in NPC metastasis. A total of 239 DEGs were identified. DEGs were mainly enriched in oocyte maturation-related pathways, cytokine-related pathways, cell cycle-related pathways, cancer-related pathways, and homologous recombination-related pathways. In addition, the top 10 nodes with the higher degree in the DEG PPI network were as follows: CDK1, CCNB2, BUB1, CCNA2, AURKB, BUB1B, MAD2L1, NDC80, BIRC5, and CENPF. The results indicated that DEGs may be involved in the pathogenesis of NPC by regulating cell cycle and mitosis, which can be used as molecular biomarkers for the diagnosis of NPC. In addition, we identified 87 DEGs with FC > 2 and *P* < 0.01 from the metastasis spectrum of NPC. The intersection gene between DEGs of NPC and normal NP tissue samples and those of the metastatic spectrum of NPC was identified to be VRK2. The expression of VRK2 in NPC samples was significantly higher than that in normal NP tissue, and similarly, VRK2 expression was significantly upregulated in metastatic samples compared with nonmetastatic samples (*P* < 0.05). Therefore, VRK2 may be a biomarker for predicting the metastasis of NPC patients after treatment.

## 1. Introduction

Nasopharyngeal carcinoma (NPC) is a malignant tumor that occurs at the top and lateral of the nasopharyngeal (NP) cavity, which is one of the most common head and neck malignancies in East Asia and Southeast Asia [1]. The pathogenesis of NPC is diverse, which may be related to viral infection, familial or genetic predisposition, and individual factors [2]. It tends to occur in areas with a high nickel content in salted products, food and water, and in patients with close relatives with NPC. Patients with NPC may not feel any symptoms in the early clinical stages. However, as the disease progresses, patients may experience symptoms such as tinnitus, hearing loss, nasal congestion, and nosebleed, as well as complications such as dermatomyositis and occult cancers of the head and neck [3]. At present, the mainstay of treatment for NPC is a comprehensive treatment model led by radiotherapy and chemotherapy [4]. With the development of radiotherapy technology and the application of comprehensive treatment modes, the treatment effect of NPC has been significantly improved. You et al. [5] reported in a multicenter phase III randomized clinical trial that the 2-year overall survival of patients with chemotherapy combined with radiotherapy was 76.4%. The treatment effect of early NPC is very significant, but due to nonspecific early symptoms and rapid disease progression, most patients are already in the local middle and late stages when they see a doctor, resulting in their loss of the best timing for treatment. In addition, some patients develop distant metastasis despite short-term remission following systemic treatment. Distant metastasis has become one of the main causes of treatment failure in cancer patients [6]. Once NPC patients develop distant metastases, the overall prognosis is poor and the cure rate is low [7]. Distant metastases are common in bone, lung, liver, and distant lymph nodes, most of which occur within 3 years after radical radiotherapy. Therefore, we explored differentially expressed genes (DEGs) in NPC tissues and screened out biomarkers that can predict metastasis in NPC patients after treatment, so as to provide guidance for the treatment of NPC.

With the completion of the Human Genome Project (HGP) and the rapid development of molecular biology-related disciplines, more and more gene animal, plant, and microorganism sequences have been determined, contributing to the rapid growth of gene sequence databases at an unprecedented rate [8–10]. The emergence as well as the constant advance in DNA chip and high-throughput sequencing (NGS) technology has made it possible to study the biological information and functions of many genes. In recent years, DNA chips and NGS have been widely used in research of life sciences and have attracted extensive attention from the scientific community [11]. Among them, Gene Expression Omnibus (GEO) is currently one of the largest chip public databases that provide data inquiries and can be submitted to the public for storage and exchange after years of creation and maintenance. It mainly collects and sorts out various expression chip data, including methylation chip, LncRNA, CNV chip, and high-throughput sequencing data [12].

The pathologic molecular mechanism of the occurrence and progression of NPC remains to be clarified, and there is still a lack of specific tumor biomarkers to predict the early diagnosis and clinical outcome of NPC. Yang et al. [13] used subtractive suppression hybridization (SSH) to isolate differential expression between metastatic 5-8F and nonmetastatic 6-10B NPC cell lines and found that in 5-8F cell lines, 20 of the 192 clones were significantly upregulated. Of the 20 clones, 16 were previously identified genes (flotilin-2, ezrin, pim-3, fli-1, mel, neugrin, znf216, ASB1, raly, UBE2A, keratin6A, TMED7, EIF3S9, FTL, two ribosomal proteins RPL21, and RPL16), and two were predicted genes (c9orf74 and MDS006). In this paper, we collected and downloaded NPC tissue-related gene expression profiles and NPC-metastasis related gene expression profile data from the GEO database and used bioinformatics and online analysis tools to perform differential expression analysis on the datasets of the GEO database. The DEGs were screened out, and the protein molecular regulatory network of the disease-related DEGs was constructed. Subsequently, functional enrichment analysis was carried out to study the mechanism of NPC occurrence, providing a theoretical basis for the diagnosis and treatment of NPC. Further analysis of the effect of DEGs on the recurrence and metastasis of NPC was performed, with the aim of identifying potentially important genetic markers and better understanding the molecular mechanism of NPC recurrence and metastasis.

## 2. Materials and Methods

### 2.1. Selection and Collection of NPC Data

The GSE61218 dataset, containing the expression profile data of NPC and normal NP tissues, was downloaded from the database GEO (https://www.ncbi.nlm.nih.gov/geo/). The data is based on the Agilent-043965 custom human array oelinc_xw test on the GPL19061 platform, including 10 specimens of NPC tissue and 6 specimens of normal NP tissue [14]. R software was used to extract gene expression profile data in the chip for subsequent data analysis.

The GSE103611 dataset with metastatic and nonmetastatic expression profile data of NPC was selected and downloaded from the GEO database. The data is based on the GPL19251 platform [HuGene-2_0-st] Affymetrix Human Gene 2.0 ST Array detection, which consists of 24 samples with distant metastases from NPC after radical resection and 24 samples without distant metastases from NPC after radical resection. Then, the downloaded probe expression profile Series Matrix File(s) file was unzipped. The limma R package was used, and the differential probes for metastasis and nonmetastasis of NPC in the expression profile were screened out with the screening conditions set as FC > 1 and *P* < 0.01. The probe was then used to match the GPL19251 platform file to get the corresponding DEGs.

### 2.2. Data Preprocessing

The downloaded probe expression profile Series Matrix File(s) file was unzipped, and the GPL19061 platform file was matched with the R language without deleting the corresponding probe. If multiple probes corresponded to the same gene, their expression values were added and the average was obtained.

### 2.3. Extraction and Screening of DEGs between NPC and Normal NP Tissues

The R software limma package [15] was used to set the filter condition as the |Fold Change| > 2 times and adjust *P* < 0.01 (FC > 2 and adjust *P* < 0.01). Adjust *P* was adjusted by the Benjamini-Hochberg method. The DEGs between NPC and normal NP tissues in the expression profile were screened out. The selected DEGs were subjected to KEGG functional enrichment analysis [16]. Functional enrichment used KOBAS 3.0 functional enrichment analysis tool (http://kobas.cbi.pku.edu.cn/kobas3/genelist/). The “pheatmap” package of R software was used to draw the expression heat map of DEGs.

### 2.4. Construction of Protein Molecular Regulatory Network of Disease-Related DEGs

In order to explore the interactions of DEGs at the protein level and establish a protein-protein interaction (PPI) network, the search tool for STRING database (http://string-db.org) was used to identify the interactions between proteins, with the comprehensive score ≥ 0.9 as the standard. Only those PPIs verified by previous experiments or coexpression analysis or recorded in the relevant database are screened out to construct the network. In addition, it is required that at least one gene in each PPI should be an identified DEG. Finally, Cytoscape version 3.7.2 was used to visualize the PPI network.

## 3. Results and Discussion

### 3.1. DEGs of NPC and Normal NP Tissue

After preprocessing the original probe expression profile, a 21748∗16 gene expression profile matrix was obtained. From 21748 genes, a total of 239 DEGs with FC > 2 and adjust *P* < 0.01 were screened. Compared with normal NP tissue, 168 genes were upregulated and 71 genes were downregulated in NPC tissue (Figure 1). The top 30 genes with most significant differences are shown in Table 1, and Figure 2 is a heat map of the top 30 DEGs.

### 3.2. Pathways for Enrichment of DEGs in NPC and Normal NP Tissues

KOBAS 3.0, the online functional enrichment analysis tool, was used, and the criterion was set as *P* < 0.05. The results showed that DEGs were mainly enriched in 6 types of pathways, namely, progesterone-mediated oocyte maturation, oocyte meiosis, and cytokine related pathways (viral protein interaction with cytokine and cytokine receptor, chemokine signaling pathway, and cytokine-cytokine receptor interaction), cell cycle related pathways (cell cycle, p53 signaling pathway, cellular senescence, human T-cell leukemia virus 1 infection, and viral carcinogenesis), cancer-related pathways (small cell lung cancer, human papillomavirus infection, and pathways in cancer), homologous recombination pathways (homologous recombination, and fanconi anemia pathway), and other pathways (platinum drug resistance, systemic lupus erythematosus, and hepatitis C), as shown in Figure 3.

### 3.3. PPI Network of DEGs in NPC and Normal NP Tissues

The PPI network was constructed by combining the DEGs with the known interactions in the STRING database (Figure 4). The top 10 nodes with the highest degree in the PPI network were CDK1, degree = 51; CCNB2, degree = 43; BUB1, degree = 42; CCNA2, degree = 39; AURKB, degree = 39; BUB1B, degree = 38; MAD2L1, degree = 36; NDC80, degree = 35; BIRC5, degree = 34; and CENPF; degree = 34. CDK1 showed the highest degree, indicating that it may play a leading role in the development of NPC.

### 3.4. DEGs between Metastatic and Nonmetastatic NPC

In NPC metastatic and nonmetastatic probe expression profiles, a total of 90 differential probes with FC > 2 and *P* < 0.01 were screened (Figure 5); 90 differentially expressed probes corresponded to 87 genes. Compared with nonmetastatic NPC patients, the 87 genes were upregulated in metastatic patients (see Table 2). The heat map of the first 30 top DEGs is shown in Figure 6.

### 3.5. The Correlation of DEGs of NPC and Normal NP Tissues with Recurrence and Metastasis of NPC

There was an intersection between the DEGs in NPC and normal NP tissues and the DEGs in NPC recurrence and metastasis (Figure 7), and the intersection gene was identified to be VRK2. The expression of VRK2 in metastatic-NPC samples was significantly higher than that in nonmetastatic NPC samples (*P* < 0.05); in addition, significantly higher VRK2 expression was found in NPC tissue samples compared with normal NP tissue samples (*P* < 0.05), as shown in Figure 8. It is suggested that VRK2, a DEG of NPC and normal NP tissue, may be involved in the metastasis of NPC.

## 4. Discussion

Previous studies have shown that there are several main factors related to the development of NPC, including dietary, carcinogenic virus infection, Epstein-Barr virus (EBV), and genetic susceptibility. Genetic changes in specific chromosomal regions, genes carrying specific cancer-related single nucleotide polymorphisms (SNPs), and epigenetic changes (promoter hypermethylation) are key factors for the development of NPC [17]. With the continuous development of radiotherapy and chemotherapy technology, the treatment of NPC has significantly improved, but there are still some patients with distant metastasis after treatment. Therefore, there is an urgent need to find new biomarkers that can predict metastasis in NPC patients after treatment.

Based on the bioinformatics analysis, this paper used the NPC chip data in the GEO database to screen out 239 DEGs between NPC and normal NP tissues. KEGG enrichment analysis showed that the DEGs were closely related to different pathways, including progesterone-mediated oocyte maturation, oocyte meiosis, viral protein interaction with cytokine and cytokine receptor, chemokine signaling pathway, cytokine cytokine receptor interaction, cell cycle, p53 signaling pathway, cellular senescence, human T-cell leukemia virus 1 infection, viral carcinogenesis, small cell lung cancer, human papillomavirus infection, pathways in cancer, homologous recombination, fanconi anemia pathway, platinum drug resistance, systemic lupus erythematosus, and hepatitis C. Of them, the p53 signaling pathway has been confirmed to be involved in the occurrence of NPC. The tumor suppressor gene p53 is closely related to the regulation of cell growth, differentiation, and apoptosis [18]. Therefore, the abnormality of p53 signaling pathway can promote the malignant proliferation of NPC cells and inhibit apoptosis. Cell cycle refers to the process a cell undergoes from the completion of one division to the end of the next division, which controls cell division and proliferation. Therefore, abnormal NPC cell cycle can enhance the malignant proliferation of NPC cells [19]. Some viruses that pose a heavy burden on humans, such as EBV, HBV, HCV, HTLV-I, HIV-1, and HPV, have been classified as primary carcinogens by the International Agency for Research on Cancer, bearing responsibility for nearly 15% of all human cancers [20]. EBV, separated from the cytoplasm by circular DNA, mainly infects human pharyngeal epithelial cells and lymphocytes and can be integrated into the chromosomes of cells. During latent infection, EBV expresses a variety of latent genes, which interact with oncogenes to cause host cell cycle disorders, thus promoting the occurrence and development of EBV-related tumors [21, 22]. In addition, the pathways related to DEGs between NPC and normal NP tissue samples studied in this study, such as oocyte meiosis, pathways in cancer, and homogeneous recombination, are closely related to the malignant proliferation of NPC cells. Our research results showed that the 239 DEGs identified in NPC and normal NP tissues were significantly related to the occurrence of NPC and may be molecular biomarkers for the diagnosis of the disease.

In order to further analyze the interactions between the 239 DEGs and proteins, we used the STRING database to find the interactions between the proteins and visualized them with Cyctoscaper software. The results showed that the CDK1 node has the highest degree, indicating that it may play a leading role in the occurrence of NPC. The protein encoded by CDK1 is the serine/threonine protein kinase family. This protein is the catalytic subunit of M-phase promoting factor (MPF), which is essential for the G1/S and G2/M transitions of the eukaryotic cell cycle [23]. The protein regulates the cell cycle by regulating the phosphorylation of target proteins [24]. It shows that DEGs may participate in the pathogenesis of NPC by regulating cell cycle.

Further, we explored the effects of the 239 DEGs in NPC tissues on the metastasis of NPC patients after treatment to identify genetic markers that can predict the metastasis of NPC. A total of 87 metastatic and nonmetastatic DEGs were identified from the NPC metastasis profile downloaded from the GEO database. The intersection gene between the DEGs between NPC and normal NP tissue samples and those of the metastatic profile of NPC was found to be VRK2. The level of VRK2 in NPC samples was significantly higher than that in normal tissue samples, and VRK2 expression was also significantly higher in metastatic samples compared with nonmetastatic samples. VRK2-encoded proteins are effectors of signaling pathways that regulate tumor cell apoptosis and growth [25]. Vázquez-Cedeira et al. [26] confirmed for the first time that human VRK2 regulated the target and function of cancer cell invasion through the NFAT pathway and COX-2 expression. Mu et al. [27] also showed that VRK2 regulated the ERK1/2/AKT signaling pathway by targeting miR-145-5p to inhibit the occurrence and development of lung adenocarcinoma. NPC is an epithelial tumor closely related to EBV infection. Li et al. [28] used a yeast two-hybrid system to screen cDNA libraries from human prepuce keratinocytes and isolated the cell gene encoding human vaccinia virus B1R kinase-related kinase 2 (VRK2). The interaction between cell VRK2 and viral BHRF1 protein was further confirmed by experiments. BHRF1 is an early gene product of EBV and is homologous to Bcl-2 in structure and function. Their results suggest that human VRK2 interacts specifically with EBV BHRF1 and that this interaction is involved in protecting cells from apoptosis. These studies show that VRK2 plays an important role in tumor metastasis, suggesting that VRK2 may be a biomarker for predicting metastasis in NPC patients after treatment, but its specific mechanism needs further experiments. The limitation of this study is that we did not conduct relevant cell biology experiments to explore the effects of VRK2 on the proliferation, apoptosis, invasion, and metastasis of NPC cells, so as to further confirm that VRK2 may be a biomarker for predicting metastasis in patients with NPC after treatment. Therefore, in the follow-up research, we will further investigate the influence mechanism of VRK2 on the proliferation, apoptosis, metastasis, and invasion of NPC cells.

## 5. Conclusion

In this paper, the expression profiles of NPC tissues and normal NP tissues (GSE61218), as well as those of distant metastatic and nonmetastatic tissues (GSE103611) of NPC after radical treatment were obtained from the GEO database for analysis. A total of 239 DEGs were identified between NPC and normal NP tissue samples. DEGs are mainly enriched in oocyte maturation-related pathways, cytokine-related pathways, cell cycle-related pathways, cancer-related pathways, and homologous recombination-related pathways. In addition, the top 10 nodes with the highest degree in the DEG PPI network were CDK1, CCNB2, BUB1, CCNA2, AURKB, BUB1B, MAD2L1, NDC80, BIRC5, and CENPF. It indicates that DEGs may participate in the pathogenesis of NPC by regulating cell cycle and mitosis, which can be used as molecular biomarkers to diagnose the disease. In addition, 87 DEGs were identified from the metastatic spectrum of NPC. The intersection gene between the DEGs of NPC and normal NP tissue samples and the DEGs of the metastatic spectrum of NPC was VRK2. The level of VRK2 in NPC samples and metastatic samples was significantly higher than that in normal tissue samples and nonmetastatic samples, indicating that VRK2 may be a biomarker for predicting the metastasis of NPC patients after treatment. However, the specific mechanism of VRK2 on the metastasis of NPC needs further experimental study.

## Figures and Tables

**Figure 1:** Gene volcano plot of genes (scattered dots) in nasopharyngeal carcinoma and normal nasopharyngeal tissues. The red dots represent DEGs (FC > 2 and adjust *P* < 0.01), the black dots represent FC < 2 (NS), the green dot represents FC > 2 and adjust *P* > 0.01 (Log2FC), and the blue dot represents FC < 2 and adjust *P* < 0.01 (*P* value). There were 168 differentially upregulated genes and 71 differentially downregulated genes.

**Figure 2:** Heat map of differentially expressed genes between nasopharyngeal carcinoma and normal nasopharyngeal tissues (top 30).

**Figure 3:** Visualized bar graph of KEGG pathway enrichment analysis of differentially expressed genes between nasopharyngeal carcinoma and normal nasopharyngeal tissues. Each row represents an enrichment function. The length of the bar graph represents the enrichment ratio, which is calculated as number of input genes/number of background genes. The colors represent different clusters.

**Figure 4:** The PPI network of DEGs. Yellow represents the top 10 nodes with the highest node degree in PPI.

**Figure 5:** Volcano plot of metastatic and nonmetastatic genes in nasopharyngeal carcinoma. The red dots represent differentially expressed genes (FC > 2 and adjust *P* < 0.01), the black dots represent FC < 2 (NS), the green dot represents FC > 2 and adjust *P* > 0.01 (Log2FC), the blue dot represents FC < 2 and adjust *P* < 0.01 (*P* value). There were 87 differentially upregulated genes.

**Figure 6:** Heat map of differentially expressed genes between metastatic and nonmetastatic nasopharyngeal carcinoma (top30). The *Y*-coordinate represents genes, and the *X*-coordinate represents the sample type; M stands for metastatic, and NM stands for nonmetastatic.

**Figure 7:** Venn diagram. The intersection of differentially expressed genes in nasopharyngeal carcinoma and normal nasopharyngeal tissues and differentially expressed genes in recurrence and metastasis of nasopharyngeal carcinoma.

**Figure 8:** (a) VRK2 gene expression in nasopharyngeal carcinoma metastatic (M) and nonmetastatic (NM) samples. The *x*-coordinate indicates sample type. (b) VRK2 gene expression in nasopharyngeal carcinoma (cancer) and nasopharyngeal normal samples (normal).

**Table 1:** Differentially expressed genes between nasopharyngeal carcinoma and normal nasopharyngeal tissues (top 30).

Gene ID	Gene symbol	logFC	AveExpr	*t*	*P* value	Adj.*P*.Val	*B*
132203	SNTN	4.73639344	4.293365	4.953732378	0.000127864	0.00376799	1.215158881
84417	C2orf40	4.446700323	3.698535231	6.523380343	5.75E-06	0.000735367	4.212762313
84740	AFAP1-AS1	-4.365093483	5.180849194	-6.826805603	3.28E-06	0.000603972	4.751506898
3627	CXCL10	-4.223607875	9.514582222	-10.11732825	1.58E-08	8.40E-05	9.727523535
6355	CCL8	-4.21263275	4.698460569	-4.925883253	0.000135465	0.003895172	1.159166643
7130	TNFAIP6	-4.202777733	5.652378	-4.73614851	0.000201197	0.004834949	0.775667901
254956	MORN5	4.068387633	3.677781363	5.782057665	2.39E-05	0.001577239	2.838908492
643037	LOC643037	3.94711914	4.127274938	4.69778847	0.000218042	0.005066441	0.697730013
127254	C1orf173	3.907480223	4.173234194	4.40528337	0.000404256	0.00722412	0.099641725
3694	ITGB6	-3.881607057	4.965139744	-5.472273919	4.43E-05	0.002132906	2.241751473
92196	DAPL1	-3.872643803	7.226308219	-4.694718751	0.000219451	0.005082659	0.691487626
92749	CCDC164	3.86936162	4.349147638	4.581909962	0.000278215	0.005823499	0.461548973
83659	TEKT1	3.815984697	3.610940581	4.174612598	0.000660784	0.009809375	-0.37568957
144448	TSPAN19	3.738657203	3.429926531	4.714003076	0.000210753	0.004987428	0.730689591
118932	ANKRD22	-3.71879161	4.242687956	-12.63708752	5.85E-10	6.36E-06	12.61846049
6373	CXCL11	-3.682313417	8.951486069	-7.466774635	1.04E-06	0.000440403	5.841971939
155465	AGR3	3.669091687	5.483890163	4.348694929	0.000455897	0.007715837	-0.016724757
339145	FAM92B	3.640374663	4.073114169	5.491501891	4.26E-05	0.002105329	2.279187714
92312	MEX3A	-3.636418297	3.589654319	-4.272620895	0.000536052	0.008584723	-0.173427076
5743	PTGS2	-3.592431193	5.143853063	-4.334413762	0.000469958	0.007880215	-0.046119862
89765	RSPH1	3.43380343	5.544439631	4.480828157	0.000344443	0.006638966	0.254690263
157313	CDCA2	-3.39596974	4.309228388	-7.952300907	4.54E-07	0.000315876	6.628084753
54443	ANLN	-3.394120193	4.771685038	-6.208386848	1.04E-05	0.000998181	3.638833759
222256	CDHR3	3.374758548	3.711877591	5.058727993	0.000102923	0.003325965	1.425525185
6752	SSTR2	-3.3575362	3.64976185	-4.569776087	0.000285425	0.005917477	0.436756759
123872	DNAAF1	3.296873622	3.324685028	4.931875416	0.000133791	0.003869275	1.17122094
51514	DTL	-3.290419287	5.410863188	-7.521102521	9.49E-07	0.000440403	5.931686769
389161	ANKUB1	3.283178657	3.992556256	4.310362856	0.000494639	0.008168123	-0.095647948
83894	TTC29	3.26978886	3.219553713	4.974128821	0.000122575	0.003683809	1.256116198
642587	MIR205HG	-3.266736417	6.798005794	-5.601522108	3.42E-05	0.001888565	2.492462545

**Table 2:** Differentially expressed genes between metastatic and nonmetastatic nasopharyngeal carcinoma (top30).

Geneid	logFC	AveExpr	*t*	*P* value	Adj.*P*.Val	*B*
RIC8B	2.375960742	3.263627651	5.76107050	5.42E-07	0.144165299	0.678651435
IDH2	2.357683596	4.150624523	5.64451065	8.17E-07	0.144165299	0.526110055
SNX13	2.799302875	4.641222412	5.21164255	3.71E-06	0.296997898	-0.047336097
IDH3B	2.657161722	3.797567709	5.17537416	4.21E-06	0.296997898	-0.095777647
DOCK5	2.007484664	2.886528683	5.08141533	5.82E-06	0.342396379	-0.221478762
SLCO3A1	2.458434397	3.667017908	4.92185196	1.01E-05	0.444089226	-0.435482949
NA	2.111329032	3.034006222	4.60661926	2.93E-05	0.794687398	-0.859113324
CPT1B	2.585729704	3.628989454	4.48504919	4.39E-05	0.841704314	-1.022330075
NCAPH2	2.524770238	4.512544922	4.31429345	7.72E-05	0.841704314	-1.250960331
FAM208A	2.060351462	4.256758085	4.09197691	0.00015876	0.841704314	-1.546776323
LUC7L3	2.051955233	3.984524328	3.93707045	0.00026007	0.841704314	-1.751082775
PLXNB1	2.366888782	4.198615236	3.92367042	0.00027132	0.841704314	-1.768669542
VGLL4	2.203890951	3.692174461	3.88673867	0.00030479	0.841704314	-1.817061539
PIKFYVE	2.069407454	3.957492054	3.85771422	0.00033385	0.841704314	-1.855008404
SQSTM1	2.704433462	6.572252601	3.82334620	0.00037173	0.841704314	-1.899841396
ESYT2	2.488310392	4.660026253	3.82245751	0.00037277	0.841704314	-1.900999208
SPICE1	2.04465473	4.369786302	3.67589374	0.00058664	0.841704314	-2.090846142
YBEY	2.196392614	7.688738652	3.65950270	0.00061684	0.841704314	-2.11193267
AGRN	2.171473709	5.673356282	3.62550519	0.00068432	0.841704314	-2.155569203
XPOT	2.284908294	3.712960018	3.62044606	0.00069495	0.841704314	-2.16205093
GNAS	2.402798764	7.475241485	3.60766363	0.00072250	0.841704314	-2.178413835
LYST	2.287754018	5.408772982	3.58526810	0.00077333	0.841704314	-2.207034049
CFP	2.354234514	6.973115353	3.57877866	0.00078868	0.841704314	-2.215315479
CD46	2.124786184	6.266164679	3.55523891	0.00084686	0.841704314	-2.245310519
MYOF	2.289126134	4.944656867	3.54021184	0.00088612	0.841704314	-2.264421025
INVS	2.21886402	5.348487784	3.53915975	0.00088894	0.841704314	-2.265757904
AKAP1	2.42526721	5.099006759	3.53681505	0.00089524	0.841704314	-2.26873676
IVNS1ABP	2.594644228	7.174776083	3.52217873	0.00093554	0.841704314	-2.287315199
MAGI1	2.571121918	5.595876999	3.51585726	0.00095347	0.841704314	-2.295330454
MYL5	2.329321318	7.096841016	3.51272355	0.00096249	0.841704314	-2.29930181

## Data Availability

The data used to support the findings of this study are available from the corresponding authors upon request.
